The article "Prognostic Significance of CCDC137 Expression and Its Association with Immune Infiltration in Hepatocellular Carcinoma" was published in 2022. Journal: Dis Markers.

# Prognostic Significance of CCDC137 Expression and Its Association with Immune Infiltration in Hepatocellular Carcinoma

**DOI:** 10.1155/2022/5638675

**Published:** 2022-08-24

**Authors:** Lu Bai, Zhao-Xu Yang, Jian-Shan Liu, De-Sheng Wang, Heng-Chao Yu

**Affiliations:** ^1^Department of Clinical Laboratory, Xijing Hospital, Air Force Military Medical University, Xian, China; ^2^Department of Hepatobiliary Surgery, Xijing Hospital, Air Force Military Medical University, Xian, China

## Abstract

Globally, hepatocellular carcinoma (HCC) is one of the most common causes of cancer-associated mortalities. The clinical outcome of HCC patients remains poor due to distant metastasis and recurrence. In recent years, growing evidences have confirmed that the coiled-coil domain-containing (CCDC) family proteins are involved in the progression of several diseases. However, the expression and clinical significance of the coiled-coil domain-containing 137 (CCDC137) in hepatocellular carcinoma (HCC) have not been investigated. Level 3 mRNA expression profiles and clinicopathological data were obtained in TCGA-LIHC. Differentially expressed genes (DEGs) were screened between 371 HCC and 50 nontumor specimens. The prognostic value of CCDC137 was analyzed in HCC patients. The correlations between CCDC137 and cancer immune infiltrates were investigated. In this study, a total of 2897 DEGs were obtained: 2451 genes were significantly upregulated and 446 genes were significantly downregulated. KEGG assays revealed that these DEGs were involved in tumor progression. Among 2897 DEGs, we found that CCDC137 expression was distinctly increased in HCC specimens compared with nontumor specimens. A high level of CCDC137 expression was related to an advanced tumor stage and grade. Moreover, patients with higher levels of CCDC137 expression had a shorter overall survival and disease-free survival than patients with lower CCDC137 levels. CCDC137 expression was positively correlated with infiltrating levels of several immune cells, such as CD8 T cells and Th2 cells. Finally, in vitro experiments confirmed that CCDC137 expression was highly expressed in HCC cells, and its knockdown suppressed the proliferation of HCC cells. Taken together, our findings revealed that CCDC137 might be used as a biomarker for immune infiltration and poor prognosis in HCC, which offered fresh insight on potential therapies for HCC.

## 1. Introduction

Hepatocellular carcinoma (HCC) is one of the leading causes of cancer-related death worldwide [1]. According to the Global Cancer Statistics, for the year 2020, there were around 906,000 newly diagnosed instances of liver cancer and approximately 830,000 deaths caused by liver cancer worldwide that year [2]. Although the majority of HCC develop in individuals who have a history of established hepatic conditions, there are a number of risk factors that are known to promote the development and progression of HCC [3, 4]. Some of these risk factors include aflatoxin B, excessive use of tobacco and alcohol, prolonged infection with hepatitis B or C virus (HBV or HCV), and exposure to iron overload [5, 6]. At the moment, surgical removal of the tumor is the recommended course of treatment for head and neck cancer caused by HCC. Despite this, the recurrence rate of HCC is still quite high, and the survival rate at five years is often less than fifty percent [7]. Therefore, it is of the utmost importance that the pathogenesis of HCC should be investigated in order to search for useful diagnostic markers and treatment targets in HCC patients.

The article "Prognostic Significance of CCDC137 Expression and Its Association with Immune Infiltration in Hepatocellular Carcinoma" was published in 2022. Journal: Dis Markers.

Characterizing prognostic factors in patients with HCC has benefited greatly from the use of transcriptome profiling, which has resulted in the generation of a number of prospective biomarkers with the potential to have clinical use [8]. However, there is a lack of consistency among different studies and the indicated signatures only provide limited predictive information. This is partially due to the small sample size and the technical variables that were used [9, 10]. An increasing number of studies, made possible by developments in gene chips and high-throughput sequencing, have demonstrated that the dysregulated mRNAs have a significant amount of potential to predict HCC prognosis [11, 12]. In addition, even though the genetic and epigenetic alterations that occur in tumor cells are essential to the progression of tumors, there is an increasing body of evidence indicating that the interaction between tumor cells and the normal cells that surround them also plays an important role in both of these processes. A complex network made up of extracellular matrix, inflammatory cells, endothelial cells, fibroblast cells, mesenchymal stem cells, and tumor cells is referred to as the tumor microenvironment (TME) [13, 14]. Over the course of the past several years, an increasing number of researches have concentrated on locating novel prognostic biomarkers implicated in the microenvironment of HCC [15]. For instance, it has been reported that CD96 showed varied levels of expression in the majority of cancerous and neighboring normal tissues. CD96 had a major impact on the prognosis of several different malignancies. Because CD96 is involved in a wide variety of immune responses, is responsible for immune cell infiltration, and influences the malignant properties of different cancers, it is a candidate for use as a biomarker in determining patient prognosis and immune infiltration in a number of different cancers [16, 17].

The article "Prognostic Significance of CCDC137 Expression and Its Association with Immune Infiltration in Hepatocellular Carcinoma" was published in 2022. Journal: Dis Markers.

In this study, we screened a novel HCC-associated gene CCDC137 which was rarely reported in previous studies. First, we presented data that CCDC137 was substantially expressed in HCC and that its upregulation was predictive of a poor prognosis for individuals with HCC. Moreover, we analyzed its association with immune Infiltration. For the purposes of this investigation, all of the data came from publicly available sources, and the analyses were carried out using Webtools and the R programming language. Our findings suggested CCDC137 as a novel biomarker for HCC patients.

## 2. Materials and Methods

### 2.1. Cell Lines and Cell Transfection

iCell (Xuhui, Shanghai, China) was the supplier of both the HCC Cells (MHCC97H, HepG2, HCCLM3, Hep3B, and SMMC-7721) and the LO2 cells which served as the control cells. RPMI-1640 served as the medium for their cultivation (with 10 percent fetal bovine serum). The cell culture condition was 37°C and 5% CO_2_. The small interfering RNAs (siRNAs) (siRNA-control and siRNA-CCDC137) were obtained from JiMa Biological Corporation (Shanghai, Pudong, China). Lipofectamine 2000 reagent kits, manufactured by Guanghua Biotech in Changsha, Hunan Province, China, were utilized in the cell transfection process. The procedure followed the guidelines included with the reagent kits.

### 2.2. Quantitative Real-Time PCR

The TRIzol reagents (Invitrogen, Carlsbad, CA, USA) were utilized in order to get the total RNA. cDNA was produced from the isolated RNA by employing the PrimeScript RT Reagent Kit (Takara, Japan) in the process of reverse transcription. Next, synthesized cDNA was subjected to RT-qPCR using the Fast SYBR Green PCR Kit (Applied Biosystems, Foster City, CA, USA) on an ABI PRISM 7300 instrument (Applied Biosystems). 2^−*ΔΔ*Ct^ method was utilized in order to calculate the fold changes in target genes. The primer sequences were presented as follows: CCDC137 5′-ACGGGGCCTATATCCACCG-3′ (forward) and 5′-CGTCGGACTTTATCTAGTCGCC-3′ (reverse); GAPDH 5′-GGAGCGAGATCCCTCCAAAAT-3′ and 5′-GGCTGTTGTCATACTTCTCATGG-3′.

### 2.3. CCK-8 Assay

Transfected HCCLM3 and MHCC97H cells were seeded at a density of 2 × 10^3^ cells per well in 96-well plates, and the plates were then incubated with RPMI-1640 media for 24, 48, 72, or 96 hours, depending on the experiment. After that, all of the cells were allowed to remain in an environment containing 10 *μ*L of CCK-8 reagents for a period of four hours. After discarding the medium, dimethyl sulfoxide was included in the experiment. After 10 minutes of shaking, a Microplate Absorbance Reader was used to measure the color reaction at 450 nm.

The article "Prognostic Significance of CCDC137 Expression and Its Association with Immune Infiltration in Hepatocellular Carcinoma" was published in 2022. Journal: Dis Markers.

## 3. Data Source

The mRNA expression patterns and the related clinical information from the patients with HCC were gathered from TCGA. This was calculated on an Illumina HiSeq RNA-seq platform, and as of March 5, 2022, the platform had 371 HCC tissues and 50 nontumorous liver tissues. Because the data from TCGA are openly and freely accessible to the public, the local ethics committees were not required to give their approval for the study.

### 3.1. Identification of DEGs between HCC and Noncancerous Tissues

The limma R package was utilized in the determination of the DEG. DEGs that had an absolute log2 fold change (FC) of more than two and an adjusted *p* value of less than 0.05 were determined to be eligible for further investigation.

### 3.2. Gene Ontology (GO) and Kyoto Encyclopedia of Genes and Genomes (KEGG) Pathway Enrichment Analysis of DEGs

The software package “clusterProfiler” of R was used to execute GO and KEGG results for visualization of the diverse genes shared by the two distinct groups of high-risk patients, and the appropriate graphs were generated afterward.

## 4. Gene Expression Profiling Interactive Analysis (GEPIA)

Further confirmation of the strongly linked genes was accomplished through the use of the internet database GEPIA (http://gepia.cancer-pku.cn/index.html). GEPIA is an interactive online database that consists of 9,736 tumor samples and 8,587 normal samples from TCGA and the GTEx projects. These projects analyze the RNA sequencing expression of the samples. In 33 distinct forms of cancer, the log-rank test and the Mantel-Cox test were used in conjunction with GEPIA to develop survival curves. These survival curves were based on gene expression and included overall survival and disease-free survival.

### 4.1. Immune Infiltration Analysis

We determined the degree of infiltration of 28 different immune cell types by using the single-sample gene set enrichment analysis (ssGSEA) method from the GSVA R package. Our calculations were based on the expression levels of genes found in 28 different published gene sets that are associated with immune cells.

### 4.2. Statistical Analysis

All statistical analyses were conducted by R (4.0.2). The significance of CCDC137 in HCC specimens and nontumor tissues was assessed by the paired Wilcoxon test. Survival curves were plotted by the Kaplan-Meier method, and the log-rank test evaluated the significance. All hypothetical tests were two-sided, and a *p* value < 0.05 was considered significant.

## 5. Results

### 5.1. Identification of DEGs in HCC

In this work, a retrospective analysis of the data was performed on a total of 371 cases with HCC and 50 specimens without tumors taken from TCGA datasets. The limma software was utilized in the analysis of the DEGs. A total of 2897 DEGs were obtained: 2,451 genes were significantly upregulated, and 446 genes were significantly downregulated (Figures 1(a) and 1(b)).

The article "Prognostic Significance of CCDC137 Expression and Its Association with Immune Infiltration in Hepatocellular Carcinoma" was published in 2022. Journal: Dis Markers.

### 5.2. Functional Correlation Analysis

Enrichment analysis using the KEGG database was carried out in order to investigate the function of DEGs. The results indicated that the 2451 upregulated genes were mainly associated with p53 signaling pathway, mRNA surveillance pathway, viral carcinogenesis, spliceosome, small cell lung cancer, and ribosome (Figure 2(a)). 446 downregulated genes were mainly associated with valine, leucine, and isoleucine degradation, tyrosine metabolism, tryptophan metabolism, steroid hormone biosynthesis, retinol metabolism, pyruvate metabolism, and PPAR signaling pathway (Figure 2(b)). Then, we performed GO assays and found that 2451 upregulated genes were mainly enriched in viral transcription, viral gene expression, spindle organization, sister chromatid segregation, ribonucleoprotein complex biogenesis, and regulation of nuclear division (Figure 2(c)). Moreover, 446 downregulated genes were enriched in xenobiotic metabolic process, steroid metabolic process, small molecule catabolic process, response to xenobiotic stimulus, organic acid catabolic process, and organic acid biosynthetic process (Figure 2(d)).

### 5.3. CCDC137 Expression Was Distinctly Increased in HCC

CCDC137 was the gene that caught our attention out of the 2,451 that were elevated. In order to determine whether or not CCDC137 expression was correlated with cancer, we analyzed its levels in a variety of tumors as well as the normal tissues. According to information obtained from TCGA database, the expression of CCDC137 was significantly increased in the majority of kinds of cancers (Figure 3(a)). In addition, CCDC137 expression was distinctly increased in HCC specimens compared with nontumor specimens (Figure 3(b)). Although data from TCGA and GTEx database did not show a distinct change of CCDC137 expression between HCC specimens and nontumor specimens, an overall trend can be observed (Figure 3(c)). After that, we investigated the relationship between the expression of CCDC137 and the clinical stages, and we discovered that a high level of CCDC137 expression was related with an advanced tumor stage and grade (Figure 3(d) and Figure 3(e)). More importantly, we found that metastasis HCC specimens showed an increased expression of CCDC137 compared with nonmetastasis HCC specimens (Figure 3(f)).

### 5.4. Correlations between CCDC137 and Prognosis

In order to investigate the possible connection between CCDC137 expression and the prognosis of HCC patients, we computed Kaplan-Meier curves for overall survival and made a comparison between those patients whose CCDC137 expression was high and those whose expression was low. The results showed that patients with higher levels of CCDC137 expression had a shorter overall survival (*p* = 5.9*e* − 06, Figure 4(a)) and disease-free survival (*p* = 0.00042, Figure 4(b)) than patients with lower CCDC137 expression levels. Based on our findings, CCDC137 might be a useful prognostic biomarker for patients with HCC.

The article "Prognostic Significance of CCDC137 Expression and Its Association with Immune Infiltration in Hepatocellular Carcinoma" was published in 2022. Journal: Dis Markers.

### 5.5. The Correlation between CCDC137 Expression and Immune Infiltration

The Spearman correlation test was used to investigate the relationship between the amount of CCDC137 expression and the amount of immune cell infiltration that was measured using single-sample sequence set enrichment analysis (ssGSEA). The expression of HTRA3 was negatively correlated with the abundance of acquired immunocytes (NK cells, cytotoxic cells, mast cells, neutrophils, DC, CD8 T cells, Th17 cells, and TReg) and positively correlated with the abundance of innate immunocytes (NK CD56bright cells, Th2 cells, and TFH) (Figure 5).

### 5.6. The Potential Roles of CCDC137 in HCC Progression

In order to verify the aforementioned findings, an aberrant expression of CCDC137 was analyzed in HCC cells using real-time quantitative PCR. As shown in Figure 6(a), we found that the level of expression of CCDC137 in five HCC cells was much higher than that that in LO2 cells. In order to investigate the role that CCDC137 plays in HCC, siRNA targeting CCDC137 was transfected into MHCC97H and HCCLM3 cells due to their relatively higher level compared with other HCC cells. CCDC137 expression in HCCLM3 and MHCC97H cells was found to be drastically reduced thanks to CCDC137 siRNA, as demonstrated by RT-qPCR (Figure 6(b)). CCK-8 data showed that the inhibition of CCDC137 expression led to a reduction in the rate of cell proliferation in HCCLM3 and MHCC97H cells (Figures 6(c) and 6(d)). These results indicate that upregulation of CCDC137 aggravated the malignancy of HCC cells.

## 6. Discussion

HCC continues to be a significant threat to public health all over the world, primarily because there are no enough reliable diagnostic tools and curative options [18]. The majority of patients identified with HCC are already in advanced stages, at which point the tumors are no longer resectable [19]. Discoveries of new biomarkers and molecular pathways have a significant clinical impact on the treatment of HCC.

Coiled-coil domain-containing (CCDC) is a structural motif that had been identified in proteins, and it exhibited an important role in a number of biological progresses, including membrane fusion, drug transport, control of gene expression, drug extrusion, and cell division [20, 21]. In addition, research has shown that the structure of the CCDC gene or the epigenetic alterations associated with it are linked to a wide variety of cancerous tumors [22]. It is believed that CCDC is involved in tumor growth and invasion of malignant tumor cells, in addition to other biological characteristics. CCDC performs a wide variety of vitally important biological functions. For instance, gastric tissues have an abundance of CCDC43 expression. Expression of CCDC43 has been linked to a number of aspects of gastric cancer, including tumor differentiation, distant metastasis, and clinical outcome of patients. The overexpression of CCDC43 in GC cells is correlated with increased rates of cell proliferation, invasion, and metastasis. It is possible for CCDC43 to upregulate and stabilize ADRM1, which would then lead to the formation of the ubiquitin-mediated proteasome [23]. In addition, Guo et al. performed pancancer analysis and identified CCDC137 as a tumor promoter and predictor of poor survivals for many tumor patients. A high level of CCDC137 has been linked to a tumor's immunosuppressive condition and has the potential to contribute to an increased infiltration of TAMs and CAFs [24]. However, the expression and function of CCDC137 in HCC have not been investigated. In this study, we discovered that the expression of CCDC137 was significantly elevated in HCC patients, and its high levels were linked to an advanced clinical stage and grade. Survival assays revealed that high CCDC137 expression was associated with shorter overall survival and disease-free survival in HCC patients. On the other hand, we also performed in vitro assays and confirmed that CCDC137 expression was distinctly increased in HCC cells. Further CCK-8 assays confirmed that CCDC137 knockdown suppressed the proliferation of HCC cells. In general, our research indicated that CCDC137 may have a role in the progression of HCC, suggesting that it may be an oncogene and underlining the fact that it may be employed as a potential biomarker and therapeutic target.

The article "Prognostic Significance of CCDC137 Expression and Its Association with Immune Infiltration in Hepatocellular Carcinoma" was published in 2022. Journal: Dis Markers.

The immunological milieu of the liver is extremely complicated because it contains a high number of innate immune cells and immune cells that behave similarly to innate immune cells [25]. It is widely held that a persistent inflammatory response is one of the primary factors that leads to the development of HCC [26, 27]. Chen et al. revealed that a favorable prognosis can be predicted by the presence of CD8+ T lymphocytes, B cells, and dendritic cells in the tumor, but a poor prognosis can be predicted by the presence of cancer-associated fibroblasts [28]. By upregulating immunological checkpoints and proinflammatory cytokines, immune cells promote the growth of tumors by allowing them to escape the body's immune system. When the immunological checkpoint is bypassed, it has been demonstrated that the host immune system is capable of producing effective antitumor immunity against tumor antigens. As a result, immunotherapy has arisen as a treatment option that can be considered for patients who have advanced HCC [29, 30]. It was indicated by our work that CCDC137 has a considerable relationship with the immune cells, particularly in NK cells, cytotoxic cells, mast cells, neutrophils, DC, CD8 T cells, Th17 cells, Treg and NK CD56bright cells, Th2 cells, and TFH. Based on our findings, CCDC137 may play a significant role in the regulation and recruitment of immune cells that infiltrate HCC.

## 7. Conclusion

Our findings suggested CCDC137 as a novel HCC-associated gene which was highly expressed in HCC. In addition, CCDC137 was found to be a useful biomarker for determining the prognosis of patients with HCC, and it was found that the expression of this biomarker has a substantial association with immune infiltrations.

## Figures and Tables

**Figure 1:** Differentially expressed genes between HCC specimens and nontumor specimens using (a) volcano map and (b) heat map based on TCGA datasets.

**Figure 2:** Results of GO and KEGG analyses. (a, b) KEGG pathway analysis in TCGA dataset. (c, d) GO analysis in TCGA dataset.

**Figure 3:** CCDC137 expression in HCC and its association with clinical progress. (a) CCDC137 expression levels in different cancer types from TCGA database analyzed. (b, c) Upregulation of CCDC137 expression in HCC samples compared with nontumor samples based on TCGA datasets and GTEx data. (d–f) CCDC137 expression was associated with clinicopathological characteristics in HCC patients, including (d) clinical stage, (e) tumor grade, and (f) nodal metastasis status.

**Figure 4:** Predictive value of CCDC137 expression for clinical outcomes in HCC patients. Survival analysis for (a) overall survival and (b) disease-free survival of HCC patients with low and high CCDC137 expressions (based on median expression) in TCGA database.

**Figure 5:** Correlation of immune cell infiltration and CCDC137 expression in HCC patients.

**Figure 6:** Knockdown of CCDC137 suppressed the proliferation of HCC cells. (a) RT-PCR for CCDC137 expression in five HCC cells and LO2 cells. (b) The expressions of CCDC137 in HCCLM3 and MHCC97H cells with its siRNA. (c, d) The proliferation of HCC cells after CCDC137 knockdown was examined by the use of CCK-8 assays. ^∗∗^*p* < 0.01.

The article "Prognostic Significance of CCDC137 Expression and Its Association with Immune Infiltration in Hepatocellular Carcinoma" was published in 2022. Journal: Dis Markers.

## Data Availability

The data used in this research are available from the corresponding authors upon reasonable request.
